# miR-339-5p Inhibits Autophagy to Reduce the Resistance of Laryngeal Carcinoma on Cisplatin via Targeting TAK1

**DOI:** 10.1155/2021/9938515

**Published:** 2021-08-03

**Authors:** Guang Li, Zexing Cheng

**Affiliations:** Department of Otorhinolaryngology-Head and Neck Surgery, The Affiliated Hospital of Yangzhou University, Yangzhou, Jiangsu 225001, China

## Abstract

Laryngeal carcinoma is a malignant disease with high morbidity and mortality. Several studies have indicated that miRNA dysfunction involves in the development of laryngeal carcinoma. In this study, the connection of miR-339-5p and laryngeal carcinoma was investigated, and qRT-PCR, CCK-8, and flow cytometry assay were used to observe the function of miR-339-5p on laryngeal carcinoma. Besides, the target database, dual-luciferase reporter assay, and western blot were used to explore the regulation mechanism of miR-339-5p on the progression of laryngeal carcinoma. The results showed that miR-339-5p was significantly downregulated in cisplatin-resistant cells of laryngeal carcinoma, and miR-339-5p upregulation could weaken the resistance of laryngeal carcinoma cells on cisplatin. Moreover, miR-339-5p could directly react with 3′-UTR of TAK1, and TAK1 could reverse the effects of miR-339-5p on the progression of autophagy. In conclusion, this study suggests that miR-339-5p can inhibit the autophagy to decrease the cisplatin resistance of laryngeal carcinoma via targeting TAK1.

## 1. Introduction

Laryngeal carcinoma is the second most prevalent malignancy of the upper aerodigestive tract, which is associated with several factors such as tobacco and alcohol consumption [1, 2]. Statistically, there are more than 13,360 new cases and 3660 deaths every year in the United States. Even with current strategies, the overall 5-year survival rate of the patients with laryngeal carcinoma is only 64.2% [3]. Moreover, more than 60% of the patients are diagnosed with advanced stage of laryngeal carcinoma when they firstly accept the diagnosis [4]. Cisplatin (DDP), an effective chemotherapy drug, has been widely used for cancer treatment in clinical practice [5]. However, the drug resistance of cancer limits the lethal effect of cisplatin on tumors [6]. Autophagy is an important tactic of cells to keep from the damages induced by starvation, oxidative stress, and poisonous substance, and increasing studies have indicated that cell autophagy is involved in the drug-resistant formation of tumor cells [7, 8].

MicroRNAs (miRNAs), a class of noncoding RNA with short chain, are responsible for transcriptional inhibition of mRNAs to regulate the expression of the related proteins in various eukaryotic cells [9, 10]. These small RNAs have been accepted as important molecular regulators in cellular life activities by many researchers [11, 12]. Many studies have demonstrated that the dysfunction of miRNAs can facilitate tumor growth, invasion, migration, and drug resistance [13]. For instance, miR-337-3p could modulate the proliferation, invasion, migration, and apoptosis of cervical cancer cells via targeting Rap1A [14]. Considering the mechanism of miRNAs, the novel therapeutic strategies have been widely used for the treatment and research of human diseases [15]. miR-339-5p has been found as a tumor suppressor to inhibit the growth of various tumors while its role in laryngeal carcinoma remains unclear [16].

In this study, we investigate the connection of miR-339-5p and laryngeal carcinoma and aimed to provide some reference for laryngeal carcinoma treatment.

## 2. Materials and Methods

### 2.1. Cell Lines and Cell Culture

Human epithelial type 2 (Hep-2) was purchased from BeNa Culture Collection Co., Ltd. (Beijing, China), and the cells were cultured with Dulbecco's modified Eagle's medium (DMEM) including 10% fetal bovine serum (FBS) purchased from Procell Life Science&Technology Co., Ltd. (Wuhan, China). The cells were cultured at 37°C in a humidified incubator with 5% CO_2_. Trypsinase solution (0.25%) (HyClone Logan, State of Utah, USA) was used to obtain adherent cells. Hep-2 cells were cultured; the cells in the culture medium contained cisplatin to establish cisplatin-resistant cells. The concentration of cisplatin was gradually increased (0.5, 1, 1.5, and 2 *μ*M). The cells were maintained in each concentration of cisplatin for a period of 3 months.

### 2.2. Cell Transfection

The miR-339-5p mimics and control miRNA were purchased from Generay Biotech (Shanghai, China). pcDNA-TAK1 and control pcDNA were also designed and purified by Generay Biotech (Shanghai, China). The cisplatin-resistant cells were seeded and cultured in 6-well plates. 4 *μ*g of DNA, 100 pmol RNA, or 10 *μ*l Lipofectamine 2000 was diluted and incubated with 250 *μ*l serum-free medium for 5 min, respectively. After that, the diluted transfectants were mixed with diluted Lipofectamine 2000 at equal proportion. The mixtures were incubated at 25°C for 20 min. The 500 *μ*l of mixtures was added in each well, and then, the cells were cultured for 24 hours.

### 2.3. RNA Extraction and RT-qPCR Analysis

The cultured cells were subjected to total RNA extraction with Trizol reagent (ThermoFisher, Massachusetts, USA). 2 *μ*g of total RNA was reverse transcribed to cDNA by the Revert Aid First Strand cDNA Synthesis Kit (Thermo Fisher, Massachusetts, USA). qRT-PCR were performed with the 7300 Real-Time PCR System (Applied Biosystems, Waltham, MA, USA). The following conditions were used: denaturation at 95°C for 3 min, followed by amplification for 40 cycles at 95°C for 12 s, at 62°C for 40 s, and at 70°C for 30 s. The relative expression levels of miRNAs were calculated with the 2^−((*ΔΔ*Ct)^ method [17, 18]. The primers of miR-339-5p and TAK1 were synthesized and purified by RiboBio (Guangzhou, China). U6 was used as the endogenous controls. The primer sequences of miR-339-5p and U6 are listed in Table 1.

### 2.4. Western Blot

The total proteins of cells were extracted with RIPA buffer and 1% PMSF (Beyotime, Shanghai, China) for western blot. The concentration of the proteins was measured using a Pierce BCA protein assay kit (Beyotime, Shanghai, China). The proteins in the extracts were separated by 15% SDS-PAGE gels and then were transferred from SDS-PAGE onto PVDF membranes. After that, the membranes were immersed into 5% fat-free milk and cultured for 1 hour. The membranes were incubated with the related first antibody of the protein at 4°C for 24 hours. Subsequently, the membranes were incubated with the second antibody for 1 hour. Finally, the relative expression levels of the proteins were observed by a chemiluminescence detection system. The antibodies were used as follow: anti-TAK1 (1 : 1000, ab10979591, ThermoFisher, Massachusetts, USA); anti-LC3B (1 : 1000, ab2234770, ThermoFisher, Massachusetts, USA); anti-p-AMPK (1 : 2000, ab2533585, ThermoFisher, Massachusetts, USA); anti-*β*-actin (1 : 1000, sc-47,778, Santa Cruz).

### 2.5. Dual-Luciferase Reporter Gene Assay

The 3′-UTR-mutant sequence and 3′-UTR-wild sequence of TAK1 were inserted into the pmirGLO luciferase reporter vectors, respectively. The vectors containing the mutant sequence and wild sequence of TAK1 were named as TAK1-mutant type (TAK1-mut) and TAK1-wild type (TAK1-wt). TAK1-mut and TAK1-wt were, respectively, cotransfected with miR-399-5p mimics or miR-NC into HEK-293T for 48 hours. Finally, the luciferase activity of HEK-293T was observed by a dual-luciferase reporter assay system.

### 2.6. Flow Cytometry Assay

The cisplatin-resistant cells were treated with trypsinase (0.25%, EDTA-free) and harvested. After washing three times with ice phosphate-buffered saline (PBS), 2 × 10^3^ cells were diluted in ice Annexin V-FITC binding buffer. Subsequently, the cells were incubated with 5 *μ*l Annexin V-FITC (10 *μ*g/ml) in the dark for 10 min. After that, 10 *μ*l of propidium iodide (PI 20 *μ*g/ml) was added into the cells. Finally, the apoptosis level of the cells was instantly observed by a flow cytometry equipment (BD Biosciences, State of New Jersey, USA).

### 2.7. CCK-8 Assay

The cisplatin-resistant cells were seeded into 96-well plates at 5 × 10^4^ cells/well. After transfection, then miR-339-5p mimic, miR-NC, TAK1 overexpression plasmid (pCMV-TAK1), and empty pCMV plasmid (NC) were transfected into the cells when their density is at 70%, and the cells were incubated for 48 hours. After that, 10 *μ*l of CCK-8 solution (Amyjet, Wuhan, China) was added to each well, and the cells were incubated for 2 hours at 37°C. Finally, a microplate reader (Flash, Shanghai, China) was used to observe the absorbance of each well at 450 nm.

### 2.8. Statistical Analysis

All assays were performed at least 3 times, independently. The results were analyzed by SPSS 20.0, and the figures were drawn by GraphPad Prism 8.0. The difference of all groups was calculated through the Chi-squared test or ANOVA with Tukey's post hoc test [19]. *P* < 0.05 meant that the difference was statistically significant [20, 21].

## 3. Results

### 3.1. miR-339-5p Was Significantly Downregulated in Hep-2 Treated with Cisplatin

To illustrate the connection of miR-339-5p and laryngeal carcinoma, the Hep-2 cells were treated with cisplatin to established cisplatin-resistant Hep-2, and the qRT-PCR was used to observe the levels of miR-339-5p in Hep-2 and resistant cells. The qRT-PCR assay reflected that the expression level of miR-339-5p was significantly downregulated in cisplatin-resistant Hep-2 cells compared with Hep-2 cells (Figure 1, *P* < 0.01).

### 3.2. miR-339-5p Upregulation Reduced the Resistance of Hep-2 Cells on Cisplatin

To further explore the functions of miR-339-5p on the progression of laryngeal carcinoma cells, the miR-339-5p mimics were transfected into cisplatin-resistant Hep-2 cells, and CCK-8, transwell, and cytometry assays were used to observe the changes of the cells. The CCK-8 assay showed that the viability of the cancer cells was effectively suppressed when transfected with miR-339-5p mimics (Figure 2(c)), *P* < 0.01). Compared with the cells in negative control groups, the apoptosis level of the cells visibly increased when miR-339-5p was downregulated (Figures 2(a) and 2(b), *P* < 0.01). Those observations suggested that the resistance of Hep-2 cells on cisplatin was inhibited when miR-339-5p was upregulated.

### 3.3. miR-339-5p Directly Target the 3′-UTR of TAK1

The databases such as miRWalk and TargetScan were used to search the potential targets of miR-339-5p. The results showed that TAK1 was a possible target of miR-339-5p (Figure 3(a)). The dual-luciferase reporter assay was used to confirm whether miR-339-5p could act with TAK1. The results showed that the luciferase activities of the cells cotransfected miR-339-5p and the wild type of TAK1 reduced significantly compared with the cells cotransfected miR-339-5p and the mutant type of TAK1 (Figure 3(b), *P* < 0.01). The luciferase activities of the cells transfected with miR-NC did not show remarkable changes. Besides, the increased expression level of TAK1 was also observed in the pathological tissues and cancer cells compared with Hep-2 cells (Figures 3(c) and 3(d), *P* < 0.01).

### 3.4. TAK1 Upregulation Reversed the Effects of miR-339-5p on Hep-2 Cells

The inhibited effect of miR-339-5p on TAK1 was proved in this study, and it was hypothesized that TAK1 is involved in the regulation of miR-339-5p on laryngeal carcinoma cells. The miR-339-5p mimics and TAK1 were cotransfected into the laryngeal carcinoma cells, and the CCK-8 and flow cytometry assay were used to observe the phenotypic changes of Hep-2 cells. The CCK-8 showed that the weakened viability of Hep-2 induced by miR-339-5p and cisplatin was reversed by TAK1 upregulation compared with the cell negative control (Figure 4(a), *P* < 0.01). Besides, the increased apoptosis level of cisplatin-resistant Hep-2 cells enhanced by miR-339-5p and was also reversed by TAK1 (Figures 4(b) and 4(c), *P* < 0.01).

### 3.5. miR-339-5p Inhibited the Autophagy Level to Reduce the Resistance of Hep-2 Cells on Cisplatin

Considering the effects of miR-339-5p on the resistance of laryngeal carcinoma, the changes of the autophagy pathway in laryngeal carcinoma cells were observed. The miR-339-5p mimics and TAK1 expressed vectors were transfected into the cells, and the western blot was used to measure the expression levels of some autophagy-related proteins in Hep-2 cells. The result showed that the increased LC3-I and reduced LC3-II in Hep-2 cells induced by miR-339-5p upregulation could be reversed by TAK1 (Figures 5(a)–5(e), *P* < 0.01). Besides, it was also found that increased miR-339-5p significantly inhibited the expression of p-AMPK when the cells suffered the impairment from cisplatin (Figure 5(f), *P* < 0.01).

## 4. Discussion

Laryngeal carcinoma poses a serious threat to the health of human. The major lethal effects of chemotherapy drugs on tumors depend on inducing the apoptosis of pathological cells [22]. Recently, increasing studies have revealed that some tumor cells can form the resistance on some antitumor drugs through the autophagy pathway [23, 24]. In this study, we illustrated the functions of miR-339-5p on laryngeal carcinoma and revealed the regulation mechanism of miR-339-5p on improving the resistance of laryngeal carcinoma on cisplatin.

Many studies have demonstrated that the dysfunction of some miRNAs contributes to the progression of tumors such as the malignant proliferation and formation of the drug resistance [25, 26]. Xu et al. [27] have found that miR-1265 was significantly downregulated in gastric cancer cells, and miR-1265 upregulation could inhibit the proliferation and induce apoptosis of the tumor cells via impairing the autophagy pathway. In this study, we found that miR-339-5p played an important role in decreasing the resistance of laryngeal carcinoma cells on cisplatin. miR-339-5p has been confirmed as a tumor inhibitor to suppress the formation and development of the tumors. Liang and Tang [28] have suggested that miR-339-5p could be negatively regulated by LINC00467, and miR-339-5p could play a tumor inhibitor role to induce the apoptosis of glioblastoma. Cisplatin, an inorganic molecular drug, has been widely used for the treatment of various cancers. It can trigger the damage of DNA via combining the nitrogen atoms of DNA base and further activate the apoptosis of tumor cells [29]. Cisplatin is one of the most effective agents, and the researches have proved that cisplatin could significantly improve the overall survival rates of the patients with cancer [30]. However, even with the satisfactory effects on tumors at the beginning of chemotherapy, the cell resistance still limits the long-term lethal effect of cisplatin in cancer treatment [31]. The program of apoptosis acts as the major mechanism on regulating the death of cells, and resistance to apoptosis is an important strategy of tumor cells away from the injury of drugs [32].

miRNAs are characterized by regulating the expression of some proteins via targeting the related mRNAs [33]. In this study, we found that miR-339-5p could directly target the 3′-UTR of TAK1, and the increased TAK1 was also observed in cisplatin-resistant cells of laryngeal carcinoma. TAK1 is a pivotal signal transducer critical for TGF-*β* functions in EMT and apoptosis via regulating the activation of the c-Jun N-terminal kinase (JNK) and p38 MAPK cascade [34]. Multiple studies have confirmed that TAK1 is related to the progressions of some tumors. TAK1 can promote the metastasis, invasion, and proliferation of tumors [35]. Iriondo et al. [36] have indicated that the abnormal expression of TAK1 is a major cause of the metastasis of triple-negative breast cancer to the lung. Besides, it has been found that TAK1 plays a key role in the drug resistance of some tumors. The results in this study showed that TAK1 upregulation could reverse the effects of miR-339-5p on depressing the cisplatin resistance of laryngeal carcinoma cells. Piro et al. have suggested that TAK1 is associated with the resistance to preoperative chemoradiotherapy of the patients with esophageal adenocarcinoma, and TAK1 can significantly reduce the apoptosis level of the tumor cells via promoting the expression of BIRC3 [37]. Moreover, we also found that miR-339-5p and TAK1 are related to the autophagy of laryngeal carcinoma cells, and miR-339-5p could inhibit the autophagy pathway way to decrease the resistance of laryngeal carcinoma on cisplatin via targeting TAK1. Autophagy is a common tactic of cells to counter the adverse factors such as starvation and poison attack. Cell autophagy is usually associated with the elevated ratio of LC3-II to LC3-I [38]. Our results showed that miR-339-5p upregulation effectively inhibits the increased ratio of LC3-II to LC3-I in cisplatin-resistant cells of laryngeal carcinoma, and the effects of miR-339-5p could be reversed by TAK1. Besides, the decreased AMPK and mTOR induced by miR-339-5p were also observed in cisplatin-resistant cells, and those phenomena could be rescued by STAK1. Therefore, this study suggests that miR-339-5p can inhibit the autophagy to improve the cisplatin resistance of laryngeal carcinoma cells via targeting TAK1.

## 5. Conclusion

In conclusion, this study suggests that miR-339-5p inhibits autophagy to reduce the resistance of laryngeal carcinoma on cisplatin via targeting TAK1.

## Figures and Tables

**Figure 1:** miR-339-5p was downregulated in cisplatin-resistant Hep-2 cells. The relative expression level of miR-339-5p was measured by qRT-PCR. ∗∗ meant *P* < 0.05.

**Figure 2:** miR-339-5p upregulation reduced the cisplatin resistance and promotes the apoptosis of cisplatin-resistant Hep-2 cells. (a, b) The effect of miR-339-5p on the apoptosis rate of cisplatin-resistant Hep-2 cells was observed by flow cytometry assay. (c) The effect of miR-339-5p on the viability of cisplatin-resistant Hep-2 cells was observed by the CCK-8 assay. ∗∗ meant *P* < 0.01.

**Figure 3:** miR-339-5p directly targeted the 3′-UTR of TAK1, and TAK1 was upregulated in cisplatin-resistant Hep-2 cells. (a) The binding effect of miR-339-5p and TAK1 was predicted by TargetScan. (b) The binding effects of miR-339-5p on 3′-UTR of TAK1 were observed by dual-luciferase reporter assay. (c, d) The relative expression levels of TAK1 in Hep-2 and cisplatin-resistant Hep-2 cells were observed by western blot. ∗∗ meant *P* < 0.01.

**Figure 4:** TAK1 reversed the effects of miR-339-5p on cisplatin-resistant Hep-2 cells. (a, b) The effect of TAK1 on the regulation of miR-339-5p on the apoptosis rate of cisplatin-resistant Hep-2 cells was observed by flow cytometry assay. (c) The effect of TAK1 on the regulation of miR-339-5p on the viability of cisplatin-resistant Hep-2 cells was observed by the CCK-8 assay. ∗∗ meant *P* < 0.01.

**Figure 5:** miR-339-3p inhibited the autophagy of cisplatin-resistant Hep-2 cells, and the TAK1 could reverse the effects of miR-339-5p on the cells. (a) The relative expression level of miR-339-5p was measured by qRT-PCR. (b–f) The relative expression levels of TAK1, LC3-I, LC3-II, and pAMPK were observed by western blot assay. ∗∗ meant *P* < 0.05.

**Table 1:** Primer sequences of miR-339-5p and U6.

Name of primer	Sequences
miR-339-5p-F	5′-GGGTCCCTGTCCTCCA-3′
miR-339-5p-R	5′-TGCGTGTCGTGGAGTC-3′
U6-F	5′-CTCGCTTCGGCAGCACA-3′
U6-R	5′-AACGCTTCACGAATTTGCGT-3′

## Data Availability

The raw data can be provided if any other qualified authors need it.
